The article "5G Converged Network Resource Allocation Strategy Based on Reinforcement Learning in Edge Cloud Computing Environment" was published in 2022. Journal: Comput Intell Neurosci.

# 5G Converged Network Resource Allocation Strategy Based on Reinforcement Learning in Edge Cloud Computing Environment

**DOI:** 10.1155/2022/6174708

**Published:** 2022-05-14

**Authors:** Xuezhu Li

**Affiliations:** Department of Information Engineering, Suzhou University, Suzhou, Anhui 234000, China

## Abstract

Aiming at the problem that computing power and resources of Mobile Edge Computing (MEC) servers are difficult to process long-period intensive task data, this study proposes a 5G converged network resource allocation strategy based on reinforcement learning in edge cloud computing environment. *n* order to solve the problem of insufficient local computing power, the proposed strategy offloads some tasks to the edge of network. Firstly, we build a multi-MEC server and multi-user mobile edge system, and design optimization objectives to minimize the average response time of system tasks and total energy consumption. Then, task offloading and resource allocation process is modeled as Markov decision process. Furthermore, the deep Q-network is used to find the optimal resource allocation scheme. Finally, the proposed strategy is analyzed experimentally based on TensorFlow learning framework. Experimental results show that when the number of users is 110, final energy consumption is about 2500 J, which effectively reduces task delay and improves the utilization of resources.

## 1. Introduction

With the continuous development of technologies such as the 5G, the amount of data in various emerging application scenarios has exponentially increased. There are more and more Internet of Things (IoT) devices in various fields such as telemedicine, smart car driving, and smart cities, so all kinds of computing are everywhere [1]. However, the existing cloud computing models are difficult to manage these large-scale computing resources and perform data analysis. This is mainly reflected in the following two reasons: First, the transfer of large-scale data to cloud computing center will improve network performance and the computing power of cloud computing infrastructure brings severe challenges [2,3]. The second is that it is difficult for cloud far away from users to meet the stringent requirements of new applications such as autonomous driving on network delay and response speed [4]. Thus, both computing services and big data sources are undergoing a shift from cloud to edge [5].

Edge computing serves as an intermediate layer between the cloud computing center and user devices. It provides computing resources to users near the edge via a high-speed network by placing the edge server close to user end [6]. Among them, the user device sends computing tasks that originally need to be sent to the cloud or executed locally to edge server for execution to achieve reasonable network resource allocation, which is called computing offloading [7]. Compared with cloud servers and local computing, edge computing can provide faster network response and have more powerful computing capabilities [8]. Therefore, computing offloading and reasonable allocation of network resources by a reasonable scheduling algorithm can help users save transmission energy consumption and improve computing efficiency [9].

In the edge computing system, for security and efficiency reasons, the edge server will not open its own computing resource configuration and idle state to each user device, so it is difficult to obtain the detailed status in the system [10,11]. Under the premise of incomplete observation system constraints, task offloading and system optimization problems become more complicated. The intelligent model represented by deep reinforcement learning is an important means to solve such problems [12]. Reference [13] developed a Multi-Agent Reinforcement Learning Network to solve the Q-learning problem based on independent learners, and designed the calculation unloading strategy in IoT through random game. However, the efficiency of resource allocation strategy needs to be further improved. Reference [14] proposed a moving edge computing (MEC) network based on blockchain, which uses blockchain to control the coverage system, and adopts adaptive strategy to generate blocks and realize high-quality resource allocation. Reference [15] used deep Q network (DQN) learning to obtain the best resource allocation scheme in IoT network. However, frequent data interaction brings high network load, which becomes the main obstacle to the training of intelligent offloading models, especially computing offloading models based on deep learning.

Traditional methods also have certain research on computing task offloading and network resource allocation: For example, reference [16] solved the task unloading problem based on differential evolution algorithm, so as to realize the efficient execution of tasks, but it requires higher network bandwidth. Reference [17] designed a random mixed integer nonlinear programming method for the intensive task unloading and resource allocation in MEC, which can realize the rational use of resources, but cannot take into account energy efficiency and service delay. Reference [18] used orthogonal and non-orthogonal multiple access methods, a resource allocation scheme considering energy consumption and efficiency in MEC is formulated, but the overall delay needs to be further reduced. Reference [19] proposed a multi-objective resource allocation method for MEC, which uses Pareto archiving evolution strategy to optimize time cost and load balancing. At the same time, it combined multi-criteria decision-making and sorting preference technology similar to the ideal solution to obtain optimal resource allocation, but 5G integration scheme is not considered.

Aiming at the problem that the large amount of data transmitted in 5G network leads to channel congestion, which affects the real-time performance and energy consumption of communication, a 5G fusion network resource allocation strategy based on reinforcement learning in edge cloud computing environment is proposed. Due to the poor learning effect of basic reinforcement learning in massive data, the proposed strategy proposes a DQN offloading strategy to solve resource allocation of 5G converged networks, which can reduce the time delay. At the same time, the system energy consumption is reduced. Finally, experimental results based on TensorFlow learning framework show that proposed strategy fully considers the time and energy consumption of local and offloading to MEC execution, and solving offloading scheme by reinforcement learning can greatly reduce delay and energy consumption. Moreover, its energy consumption is about 2500J, the time delay does not exceed 7s. DQN has self-learning ability, which continuously learns during the training process to improve the accuracy of decision-making. Therefore, it can effectively reduce load and broadband utilization rate.

## 2. System Scenario and Optimization Goal

### 2.1. System Scenario

The system scenario is shown in Figure 1, consisting of *N* users, *M* base stations, and multiple MEC servers. Among them, each user is associated with the nearest base station through the wireless link and sends a task request to it. At the same time, each base station is equipped with an MEC server with multiple CPU cores. Therefore, MEC server can process the computing tasks of different users in parallel. It is assumed that user computing tasks are processed by an MEC server, regardless of situation in which computing tasks are forwarded between MEC servers.

Divide the system running time dimension into a number of time slots, and use *T*={0,1,2⋯} to represent the set of time slots for network operation, where the time length of each time slot *t* is defined as *τ*. It is assumed that most of the computing tasks of user can be processed and completed in one time slot. Due to the large amount of data, some computing tasks are divided into subtasks for processing [20]. Considering the randomness of task arrival, a two-level queue model is designed to describe the state of computing tasks, namely the user task queue model and MEC server task queue model.

### 2.2. Task Generation Model

In MEC model, it is assumed that the time interval for mobile users to generate tasks obeys Poisson distribution, and user *n* generates *k*_*n*_ mutually independent tasks, which are defined as *K*_*n*_={1,2, ⋯, *k*_*n*_}. The attribute of task *i* is defined as *φ*_*i*_={*id*_*n*_, *id*_*i*_, *sub*_*i*_, *d*_*i*_, *c*_*i*_, *l*_*i*_, *mem*_*i*_, *cpu*_*i*_}, where *id*_*u*_ represents the identity (id) of user *n* who generated task *i*, *id*_*i*_ represents the id of task, and *sub*_*i*_ represents the time when the user submits the task. *d*_*i*_ (bits as a unit) represents the amount of task data, *c*_*i*_ (CPU revolutions/bit as a unit) represents the number of CPU revolutions required to calculate one bit of task data, and *l*_*i*_=*d*_*i*_*c*_*i*_. *mem*_*i*_ and *cpu*_*i*_, respectively represent the memory and CPU resources required by computing tasks. Users are mobile and may be located near different base stations at different points in time. Thus, tasks generated by same user may be offloaded to servers in different base stations for processing.

### 2.3. Calculation Model

#### 2.3.1. Local Calculation Model

Mobile users themselves have certain computing capabilities. If the user has sufficient computing resources, then tasks can be processed locally. The computing power of local device *n* is represented by CPU frequency, which is defined as *f*_*n*,*l*_. The processing time of task on local calculation model only considers the calculation time. Therefore, the local processing time of task *i* generated by user *n* is defined as

(1) $$\begin{array}{c} t_{i,n}=\frac{l_{i}}{f_{n,l}}. \end{array}$$

The power and energy consumption of task *i* processed locally by user *n* are, respectively, defined as

(2) $$\begin{array}{c} \left\{\begin{array}{c} P_{i,n}=\gamma {\left(f_{n,l}\right)}^{3}\\ E_{i,n}=\gamma {\left(f_{n,l}\right)}^{2}l_{i} \end{array}\right), \end{array}$$

where *γ* is the effective switch capacitance.

#### 2.3.2. Edge Computing Model

Due to the insufficient computing resources of local devices, a large number of tasks generated by users cannot be processed on local computing model, but some tasks need to be offloaded to edge computing model for processing [21]. When the task is executed on MEC, the transmission time and calculation time need to be considered, and the amount of data returned by the task is very small, so the transmission time does not consider the time-consuming of result return. Before calculating the transmission time, first define the transmission rate from user device *n* to base station *m* as

(3) $$\begin{array}{c} v_{n,m}=B\;\log_{2}\left(1+\frac{p_{n}h_{n,m}}{\delta_{0}B}\right), \end{array}$$

where *B* is the communication bandwidth; *p*_*n*_ is the transmission power of user *n*. *δ*_0_ is the noise power spectral density of base station *m*; *h*_*n*,*m*_ is the channel gain between user *n* and base station *m*.

The he time for task *i* generated by user device *n* to be offloaded to server *j* of base station *m* for processing is defined as

(4) $$\begin{array}{c} t_{i,off}=\frac{d_{i}}{v_{n,m}}+\frac{l_{i}}{f_{m_{j}}}, \end{array}$$

where *f*_*m*_*j*__ is the CPU frequency of server *j* on base station *m*.

Same as time-consuming calculation, the energy consumption of task *i* generated by user *n* and offloaded to server *j* of base station *m* for processing is defined as

(5) $$\begin{array}{c} E_{i,off}=p_{n}\frac{d_{i}}{v_{n,m}}+d_{i}e_{m_{j}}, \end{array}$$

where *e*_*m*_*j*__ is the energy consumption required to calculate one bit of data.

### 2.4. Optimization Goal

The optimization goal is to reduce the average response time and total energy consumption of tasks in MEC environment, improve user service quality and save system energy cost [22]. The execution of tasks on computing nodes will be constrained by some network hardware environments [23]. Suppose that the maximum number of tasks that can be executed in parallel on the computing node is Γ, if the number of tasks is less than Γ, new tasks can be received; Otherwise, you need to wait for the resource release task to be executed. In addition, a new task can be processed only when the network resource required by the executing task and the new task is less than the total resources. The mathematical expression of the objective optimization problem is as follows:

(6) $$\begin{array}{c} \left\{\begin{array}{c} \underset{\left\{q\right\}}{\min}\bar{T}\;an\;d\;E_{total}\\ \bar{T}=\sum_{k=1}^{K}\frac{{\hat{T}}_{i}}{k},{\hat{T}}_{i}=T_{i}^{\infty }-sub_{i}\\ E_{total}=\sum_{i=1}^{k_{n}}E_{i} \end{array}\right),\\ s.t.\;q\leq \Gamma ,\\ \sum_{i=1}^{q}mem_{i}\leq C_{1},\\ \sum_{i=1}^{q}cpu_{i}\leq C_{2}, \end{array}$$

where *q* is the number of simultaneous tasks, and *C*_1_ and *C*_1_ are memory and CPU capacity respectively, and *T*_*i*_^*∞*^ is the completion time of task *i*, $E_{i}=\left\{\begin{array}{c} E_{i,n},local\;computing\\ E_{i,off},offloa\;di\;ng\;computing \end{array}\right)$.

## 3. Solutions Based on Deep Reinforcement Learning

### 3.1. Markov Decision Process Modeling

The Markov decision process is described by quadruple 〈*S*, *A*, *ψ*, *R*〉:

1. *S* is the system state collection. For an incomplete observation system, the set used by edge server to describe the system state only includes the basic information of edge server: *S*={*S*_1_, *S*_2_, ⋯, *S*_*J*_}. Among them, let *S*_*J*_ be a 5-tuple.
2. *a*_*n*_^*t*^ ∈ *A* is a finite set of actions, that is, the action of calculating offloading. The set includes the user who decides to uninstall at time *t*, and the user's action at time *t* is recorded as *a*_*n*_^*t*^. When *a*_*n*_^*t*^=0, user *n* executes locally. When *a*_*n*_^*t*^=1, user *n* offloads the task to the MEC.
3. *ψ* is the state transition matrix, and *ψ* corresponds to the mapping of *S* × *A* × *S*⟶[0,1]. That is, the probability of transitioning to next state after the end of state **S**, after the execution of action **A**.
4. *R* is the reward function. When the user needs to uninstall, the uninstall action will get a positive reward. When the decision makes system overload, a negative reward, or penalty, is given.

Reinforcement learning obtains rewards through reward function *r*_*t*_ at time *t*. For some observable system environments, the remote server can only obtain information about tasks that have been offloaded to the remote [24,25]. Therefore, it is considered that the amount of calculation saved is regarded as a reward for an offloading behavior. In order to better master the use of system resources, a punitive reward will be set. The punitive reward is set to the negative value of absolute value of current system reward, which ensures that the punitive reward value is always negative [26,27]. The punitive reward is expressed as

(7) $$\begin{array}{c} {\bar{r}}_{t}=-\left|r_{t-1}\right| \end{array}$$

Markov process corresponds to a sequence of system state transitions, that is, a trajectory sequence Ξ=〈*s*^0^, *a*^0^, *s*^1^, *a*^1^, ⋯〉 containing states and actions can be obtained. Strategy *π* corresponds to the mapping of *S* *×* *A* ⟶ [0, 1]. Deep reinforcement learning maximizes the cumulative reward expectation of Ξ during the training process to find optimal strategy *π*.

### 3.2. DQN-Based Offload Strategy

The training process based on DQN offloading strategy is shown in Figure 2.

According to the above figure, the pseudo code of algorithm based on DQN offloading strategy is shown in Algorithm 1.

Based on DQN algorithm, two neural network structures, the current Q-value network and target Q-value network are used. The two have the same neural network structure, but the parameters of their respective structures are different. The definition *θ* represents the parameters of current Q-value network, and *θ*′ represents the parameters of target Q-value network. DQN algorithm fits the action value function *Q*(*s*_*t*_, *a*_*t*_; *θ*) through Q-value network with parameter *θ*, which is calculated as follows:

(8) $$\begin{array}{c} Q\left(s_{t},a_{t};\theta \right)=E\left[\sum_{t}\chi_{t}R\left(s_{t},a_{t}\right)|s,a\right], \end{array}$$

where *χ* ∈ [0,1] is the reward discount factor.

Then select the optimal action based on value of each action generated by Q-value network:

(9) $$\begin{array}{c} a_{t}=\arg\underset{a}{\max}Q\left(s,a;\theta \right). \end{array}$$

In order to avoid not selecting the optimal local optimal solution when selecting an action, *ε*-greedy strategy is used to select an action. That is, an action is randomly selected with a small probability of *ε*, and the optimal action is selected according to (10) with a probability of 1− *ε*, so as to obtain the reward value *r*_*t*_ and next state *s*_*t*+1_. Then put quadruple (*s*_*t*_, *a*_*t*_, *r*_*t*_, *s*_*t*+1_) into the experience replay library, and sample a batch of (*s*_*t*_, *a*_*t*_, *r*_*t*_, *s*_*t*+1_) into the neural network for training. When action *a*_*t*_ is executed, the Q-value corresponding to action space *a*_*t*_ is updated, according to Bellman formula:

(10) $$\begin{array}{c} Q\left(s,a;\theta \right)=R\left(s,a\right)+\chi \underset{a^{\prime }}{\max}Q\left(s_{t+1},a^{\prime };\theta^{\prime }\right). \end{array}$$

Then minimize Loss function to update the parameters of current Q-value network. Loss function represents the predicted value of square error loss between the current Q-value network and target Q-value network. The smaller the value, the better the neural network is optimized. Generally expressed as

(11) $$\begin{array}{c} L\left(\theta \right)\approx E\left\lfloor {\left(r_{t}+\chi \underset{a^{\prime }}{\max}Q\left(s_{t+1},a^{\prime };\theta^{\prime }\right)-Q\left(s_{t},a_{t};\theta \right)\right)}^{2}\right\rfloor . \end{array}$$

Then the target *Q*-value network is updated with a delay.

## 4. Experiment and Analysis

The platform used in the experiment is Python 3.6, and Tensorflow GPU 1.14 is used for in-depth learning and optimization training. Meanwhile, the simulation parameter settings are shown in Table 1.

In addition, the proposed strategy is compared with reference [13], reference [18], and reference [19] to demonstrate its advantages. Among them, reference [13] proposed a Multi-Agent Reinforcement Learning Algorithm for computing offload of Internet of things edge computing network; Reference [18] formulated a resource allocation strategy based on orthogonal and non-orthogonal multiple access schemes; Reference [19] uses Pareto archive evolution strategy to achieve multi-objective resource allocation.

### 4.1. Analysis of Energy Consumption Results

The relationship between the number of users and energy consumption for the four strategies is shown in Figure 3.

It can be seen from Figure 3 that the energy consumption of each strategy basically shows an upward trend. However, the rise of proposed strategy has slowed down. When the number of users is 110, the final energy consumption is about 2500J. This is because too many users lead to full load of edge computing nodes, so tasks are offloaded to higher-performance cloud data centers, keeping the energy consumption of proposed strategy to a low level. Besides, it comprehensively considers local and offloading energy consumption using DQN to obtain the optimal offloading plan, which can effectively reduce energy consumption. In reference [13], although multi-agent reinforcement learning algorithm is used to obtain the optimal offloading plan, the cloud data center is not considered, so the energy consumption is increasing rapidly. The other two strategies are difficult to handle increased number of users, and the energy consumption is higher, exceeding 3500J.

### 4.2. Analysis of Time Delay Results

Similarly, the relationship between users and time delay under the four strategies is shown in Figure 4.

It can be seen from Figure 4 that reference [18] preferentially chooses to execute tasks locally to meet the requirements of delay-sensitive tasks. If the computing resources are insufficient, it will turn to high-level devices for offloading, so the delay is almost the lowest, no more than 5s. However, the strategy in reference [19] tends to preferentially offload tasks to edge nodes, and the increase in the number of users will reasonably uninstall some tasks, because the computing resources of edge nodes are in short supply and need to be queued for use, the delay will increase suddenly. As the number of users further increases, tasks are reasonably offloaded, which can alleviate time delay to a certain extent. But because of transmission link, although there is no need to queue up, a lot of time is lost in the transmission process. Even if the task continues to increase, time delay will stabilize in a higher range, about 17s. However, the delays of reference [13] and proposed strategy are relatively stable. The proposed strategy fully considers the time and energy consumption of local and offloading to MEC execution, and solving offloading scheme by reinforcement learning can greatly reduce delay.

### 4.3. Analysis of Load Balancing Rate Results

Figure 5 shows the relationship between users and load balancing ratios under the four strategies.

It can be seen from Figure 5 that the overall load balancing ratio of reference [18] strategy is relatively high. This is because it focuses on local execution, and task offloading starts from the device with the lowest performance, so as long as the device performing the task is almost fully loaded. Although some pressure was shared between 30 and 70 by offloading to edge nodes, the resources of edge nodes were quickly occupied. However, the strategy in reference [19] tends to be offloaded to MEC server, so the load balancing rate is low. This can maintain a high utilization rate for a relatively large number of edge node clusters with moderate performance. Reference [13] used multi-agent reinforcement learning algorithms for task offloading, but the load balancing rate is low. However, the algorithm performance still needs to be improved compared with DQN, so the load balancing rate of proposed strategy is the lowest, about 0.23. Reasonable utilization of users, MEC and cloud center can greatly reduce the load balancing rate.

### 4.4. Impact of Different Similarity Measurement Methods on Algorithm Execution Efficiency

According to the pipeline model, bandwidth resource bottleneck is the first dilemma faced in the offloading process. Ensuring the effective use of bandwidth resources, rather than blindly offloading too many tasks, is the key to rational use of system resources. With the increase in the number of users, the four strategies are shown in Figure 6 for network and server usage.

It can be seen from Figure 6 that compared with other strategies, the broadband utilization rate and computing resource utilization rate of proposed strategy is relatively low. Among them, the broadband utilization rate is always between 0.1 and 0.3, and computing resource utilization rate is roughly between 0.2 and 0.45. Since the proposed strategy always occupies a lower bandwidth in the decision-making process, DQN strategy is used to reasonably offload computing tasks, thereby avoiding bottlenecks in network transmission. At the same time, because fewer broadband resources are occupied, higher revenue can be obtained for servers. Reference [13] performed computational offloading based on multi-agent reinforcement learning algorithm. Although the task offloading can be completed well, MEC server has a higher requirement for computing power, so it occupies more computing resources. Reference [18] and reference [19] lacked high-performance processing algorithms and cannot balance task offloading. Thus, the broadband utilization rate and computing resource utilization rate fluctuate greatly and are at a high value.

## 5. Conclusion

With the rapid development of IoT and 5G technology, a series of new applications with computationally intensive and delay-sensitive features such as virtual reality, augmented reality and face recognition continue to emerge. In order to solve the problem of insufficient local computing power, the proposed strategy offloads some tasks to the edge of network, and builds a mobile edge system model with multi-MEC server and multi-user. This model improves the task processing capability of system by solving goal of minimizing. Besides, DQN strategy is used to obtain an offloading plan that minimizes the average response time of system tasks and total energy consumption, so as to allocate computing resources reasonably.

The proposed strategy has certain value and significance for theoretical research and practical application. However, due to resource constraints such as mobile devices, servers and base stations, experiments can only be carried out in a simulated environment that is as close to the actual situation as possible. In the future research work, we will further consider conducting physical experiments in a real environment to provide solutions to practical problems.

## Figures and Tables

**Figure 1:** System scenario.

**Figure 2:** Training process offloading strategy based on DQN.

**Figure 3:** Comparison of energy consumption of different strategies.

**Figure 4:** Comparison of time delay of different strategies.

**Figure 5:** Load balancing rate of different strategies.

**Figure 6:** Changes of network and server load with the number of users. (a) Bandwidth usage percent. (b) Computing resources usage percent.

**Algorithm 1:** Pseudo code of offloading strategy based on DQN.

**Table 1:** Experimental parameter and hyperparameter setting.

Parameter	Value
*c*_*i*_ (Cycles/bit)	500
*f*_*n*,*i*_ (GHz)	Unif (0.5.1.0)
*f*_*m*,*j*_ (GHz)	Unif (5.0,10.0)
*p*_*n*_ (mW)	150
*C* (%)	150
*D*_*n,m*_ (m)	randint (50,200)
*C*_1_ (GB)	32
*δ*_0_ (dBm/Hz)	−175
Ω	12
*χ*	0.7

## Data Availability

The data used to support the findings of this study are included within the study.
